# Efficacy and Safety Analysis of Phloroglucinol in Combination with Oxytocin for the Induction of Labor in Women with Term Premature Rupture of Membranes (PROM)

**DOI:** 10.1155/2022/2617075

**Published:** 2022-05-27

**Authors:** Jiazheng Yu, Lili Chen, Xia Wang, Xiangzhi Li

**Affiliations:** ^1^Department of Obstetrics, Taizhou Hospital of Zhejiang Province Affiliated to Wenzhou Medical University, Taizhou, 317000 Zhejiang, China; ^2^Department of Gynecology, Taizhou Hospital of Zhejiang Province Affiliated to Wenzhou Medical University, Taizhou, 317000 Zhejiang, China

## Abstract

**Objective:**

The purpose of this study was to investigate the efficacy and safety of phloroglucinol in combination with oxytocin in the induction of labor in women who had experienced term premature rupture of membranes (PROM).

**Methods:**

Data from 100 women who experienced PROM between December 2020 and December 2021 were retrospectively evaluated in this study. The puerperae were categorized into observation and control groups based on their uterine contraction regimens. The observation group consisted of 53 participants that had been treated with phloroglucinol in combination with oxytocin, and the control group consisted of 47 participants that had been treated with oxytocin alone. It was observed and compared in terms of the Bishop score before and after the administration of the puerpera to see which group had the best index. A study was performed after the drug was administered to examine its effects on the duration of labor (including the first, second, and third stages of labor), the mode of delivery (including natural vaginal delivery and cesarean section), the incidence of adverse pregnancy outcomes (fetal distress and neonatal asphyxia), successful labor induction, and complication rates.

**Results:**

Patients in the observation group had a significantly higher Bishop score after administration than those in the control group (*P* < 0.05), although there was no difference between the two groups before administration. In comparison to the control group, the observation group had a significantly higher efficacy rate for drug administration (*P* < 0.05), as well as a significantly lower occurrence of the first stage of labor (*P* < 0.05), a higher rate of vaginal natural delivery and successful induction of labor (*P* < 0.05), and a significantly lower incidence of adverse pregnancy outcomes and complications (*P* < 0.05).

**Conclusion:**

In conclusion, the use of phloroglucinol in combination with intravenous oxytocin in the process of promoting cervical ripening and induction of labor for women with PROM who are at term was investigated. This study could help women speed up cervical dilation, improve the cervical Bishop scores, shorten the total labour process, improve the effective rate of vaginal delivery, and be very safe, making it a good candidate for clinical promotion and application.

## 1. Introduction

Labor, also known as human parturition, is a physiological condition that results in the birth of a baby, the delivery of the placenta, and the signal for the initiation of lactation. It is a really difficult process [1]. If the labor is prolonged (more than 12 hours), the active laboring women become exhausted. Consequently, maternal issues like infection and excessive bleeding may develop, while fetal abnormalities such as fetal distress and asphyxia may occur [2]. Most commonly, interventions in the laboring process to shorten the time are made by rupturing membranes, using drugs to speed up contractions, and providing constant care [3, 4].

The contraction of the uterus and the effacement of the cervical cavity are the two most important characteristics of labor. If the cervix remained rigid despite intense contractions, the labor will be unable to proceed. Throughout the history of childbirth, a variety of procedures have been employed to expedite the laboring process [4]. Antispasmodic drugs are the most commonly used drugs to decrease the time of labor [5]. These drug works either by relaxing the muscles directly or by interfering with the signals sent by the nerves to the muscles that contract during labor.

The primary function of fetal membranes in pregnant women is to produce enough amniotic fluid to protect the fetus from the uterus throughout normal development. Premature rupture of membranes (PROM) refers to the rupture of fetal membranes before delivery, which causes an increase in intra-abdominal pressure in pregnant women, resulting in uneven pressure in the anterior amniotic sac and several undesirable consequences such as premature birth or dystocia [6]. PROM is closely associated with maternal gestational age, and it is more prevalent after 37 weeks of gestation. It can easily lead to infection, and if not treated in a timely and appropriate manner, it can endanger the life of the fetus [7, 8]. Therefore, if PROM occurs with an immature cervix during a maternal pregnancy of less than 37 weeks, appropriate measures should be performed to induce labor.

In clinical practice, oxytocin is frequently administered to PROM women to increase the frequency of uterine contractions. However, irregular uterine contractions may occur during the process of labor induction, resulting in a cervical spasm that prevents the expansion of the cervix during the birthing process [9]. Although the use of atropine, diazepam, and racemic anisodamine hydrochloride in obstetrics clinics was found to be effective in alleviating and promoting cervical ripening, edema, and cervical spasm to a certain extent, it was observed that these drugs are frequently associated with changes in the respiratory and circulatory systems of mothers and infants and that there are potential side effects to the use of these drugs [10, 11]. Therefore, the development of a safe and effective strategy for increasing cervical ripening is a clinical concern that must be addressed immediately in the clinical context.

Phloroglucinol is a myotropic antispasmodic drug that acts directly on the smooth muscle of the genitourinary tract and the gastrointestinal tract while having little impact on normal smooth muscle [12]. It has been extensively employed in recent years to enhance cervical ripening and softening, with promising outcomes [13, 14]. However, more studies are required to determine the efficacy and safety of its combined oxytocin in the induction of labor with the term PROM.

In this study, 100 women with PROM were chosen as the research subjects and the efficacy and safety of phloroglucinol combined with oxytocin in labor induction with term PROM were thoroughly analyzed, to provide additional evidence to support the clinical delivery plan for women with PROM.

## 2. Materials and Methods

The study population included a total of 100 women. A comparative study was conducted between patients comprising two groups (observation and control) based on their uterine contraction regimens. The observation group consisted of 53 participants that had been treated with phloroglucinol in combination with oxytocin, and the control group consisted of 47 participants that had been treated with oxytocin alone. The Bishop score was determined between two groups to see which group had the best index. Similarly, the duration of labor, the mode of delivery, the incidence of adverse pregnancy outcomes, successful labor induction, and rates of complications were all determined after the administration of combined medication in the observation group and treatment with oxytocin alone in the control group.

### 2.1. Clinical Information

The case data of 100 women with PROM who were diagnosed between December 2020 and December 2021 weeks were retrospectively analyzed. The puerperae were separated into two groups based on the different uterine contraction regimens used: the observation group, which included 53 cases (treated with phloroglucinol in combination with oxytocin), and the control group, which included 47 cases (treated with oxytocin alone). Parturients had to meet the following criteria: they must meet the clinical diagnostic criteria for term PROM, which were confirmed by B-ultrasound and laboratory tests; they must be between the ages of 20 and 35; they must have complete information and normal consciousness to participate in the study; they must be able to cooperate with the study. The following are the exclusion criteria for the investigation: parturients with mental illness, illiteracy, or communication disorder were excluded; parturients who were allergic to the medications employed in the present study were excluded; parturients with abnormal amniotic fluid, fetal heart rate, and placenta were excluded; parturients with a history of cervical surgery were excluded; parturients with liver and kidney disease, severe obstetric complications, and cardiovascular disease; parturients who do not cooperate with the research are excluded. Informed satisfaction letters were signed by all parturients indicating their consent to participate in the research. The present assessment has been confirmed by the ethics committee of Taizhou Hospital of Zhejiang Province, which is affiliated with the Wenzhou Medical University and complies with the Helsinki Declaration.

### 2.2. Treatment Methods

The control group was given an intravenous drip of 500 mL of sodium chloride injection (0.9%) and 2.5 U of oxytocin (Shanghai Harvest Pharmaceutical Co., Ltd., Shanghai, China, SFDA Approval No. H31020850). The observation group received 80 mg of phloroglucinol (Nanjing Hencer Pharmaceutical Co., Ltd., Nanjing, China, SFDA Approval No. H20046766) combined with 500 mL of sodium chloride injection (0.9%) and 2.5 U of oxytocin during labor. The infusion rate of both groups was adjusted to 8 drops/min at the beginning, and the fastest infusion rate was controlled at 40 drops/min. The concentration and rate of infusion were maintained in the presence of effective uterine contractions, for instance at an interval of 2-3 min, for a duration of 40-60 s, and at a pressure of 50-60 mmHg. An examination of the vaginal cavity was performed regularly during the therapy period to assess cervical enlargement and the descent of the fetal head.

### 2.3. Observation Indexes

(1) The Bishop scores of the two groups were compared before and after treatment [15]. The higher the score, the more cervical ripeness there is (with a total score of 13). (2) The Bishop score was used to compare the effects of two groups of puerperae after medication, and specific evaluation criteria were as follows: the cervical Bishop score of the puerpera increased by ≥3 after 12 hours of medication was considered markedly effective, increased by 1-2 after 12 hours of medication was considered effective, and that did not change was considered invalid; total effective rate = (markedly effective + effective) number of cases/total number of cases × 100%. (3) We compared the time of labor in two groups, comprising the first, second, and third stages of labor. (4) Two groups were compared regarding their delivery methods, which included vaginal and cesarean sections (5) The incidence of adverse pregnancy outcomes was compared between two groups of puerperae, which included fetal distress and neonatal asphyxia. (6) The success rates of labor induction of two groups were compared, and the criteria for success and failure of labor induction were as follows [16]: a woman with PROM at term labor induced successfully within 24 hours means the success of the induction of labor; a woman who failed to deliver under the same circumstances within 24 hours means the failure of labor induction. (7)The incidence of complications, such as cervical edema, postpartum hemorrhage, and cervical laceration, was compared between the two groups in this study

### 2.4. Statistical Analysis

The statistical analysis of the data employed was carried out using SPSS19.0 (IBM) and GraphPad Prism 8 was used to generate the experimental images. The Chi-square test (*χ*^2^) was used to analyze the number of cases as well as the percentage (%) of enumeration data. The mean ± standard deviation was used to analyze measurement data. The Student *t*-test and the LSD/t test were used to analyze differences among groups and comparisons at different time points, followed by a post-hoc test. *P* values less than 0.05 were considered statistically significant.

## 3. Results

### 3.1. Comparison of General Information

There was no significant difference in age, BMI, or childbearing history between the two groups (*P* > 0.05). The data is shown in Table 1 of the study.

### 3.2. Comparison of Bishop Scores before and after Drug Administration between Two Groups

The cervical bishop scores were evaluated before and after administration in both observation and control groups. The cervical Bishop score before administration in the observation group was 3.14 ± 0.34, while the cervical Bishop score in the control group was 3.1 ± 0.23, indicating that there was no significant difference in the cervical Bishop score between the two groups (*P* > 0.05). While the cervical bishop scores after administration in the observation group were 7.82 ± 0.36, they were found to be 6.06 ± 0.28 in the control groups, demonstrating that after administration, the scores in the observation group were significantly higher compared to the control groups (*P* < 0.05). The higher value of the bishop score indicates that the current finding is considered to be favorable for induction. The results of the study are illustrated in Table 2.

### 3.3. Comparison of Therapeutic Efficacy between Two Groups

Following administration, the number of parturients whose therapeutic efficacy was evaluated as significantly efficacious, effective, and ineffective in the group of observation was 32, 19, and 2, respectively, with an effective rate of 96.23%. As well as those of the control group, were 22, 12, and 13 correspondingly, and the effective rate was 72.34%, demonstrating that the effective rate of the observation group was significantly higher compared to the control group (*P* < 0.05). Elaborated information was demonstrated in Table 3.

### 3.4. Comparison of Labor Process between Two Groups

We compared the time of labor in two groups, comprising the first, second, and third stages of labor. The time of the first stage of labor in the observation group was shorter compared to the control group (*P* < 0.05), while no marked difference was presented for that between the second stage of labor and the third stage between the two groups (*P* > 0.05). In the observation group, however, a slightly greater change was observed in the rate of the second and third stage of labor than in the control group, indicating that overall labor stages in the observation group were shorter than in the control group, with the first stage of labor being the most obvious and displaying the most significant differences between the two groups, as displayed in Table 4.

### 3.5. Comparison of Delivery Mode between Two Groups

The vaginal delivery and cesarean section modes were compared between the two groups. 35 participants had experienced a 74.47% vaginal delivery rate out of 47 in the control group (35/47), whereas the vaginal delivery rate of the observation group was determined to be 92.45% for the 49 participants out of 53 (49/53). The finding showed a markedly higher rate of vaginal delivery when treated with the combined medication in the observation group than in the control group (*P* < 0.05), as illustrated in Figure 1.

### 3.6. Comparison of the Incidence of Adverse Pregnancy Outcomes between Two Groups

The number of neonates with fetal distress and neonatal asphyxia in the observation group was 2 and 3, respectively, and the overall incidence of adverse pregnancy outcomes was 9.43%; however, the number of neonates with fetal distress and neonatal asphyxia in the control group was 6 and 7, with a total incidence of adverse pregnancy outcomes of 27.66%, outranking the observation group in terms of incidence of adverse pregnancy outcomes (*P* < 0.05), suggesting that the combined medication was safer. The findings of the investigation are presented in Table 5.

### 3.7. Comparison of the Success Rate of Labor Induction between Two Groups

Two groups were compared for the success rate of labor induction following the administration of combination medicine. The success rate of labor induction was determined to be 94.34% in the observation group for 50 participants out of 53 (50/53), whereas the rate in the control group was determined to be 70.21% for 33 participants out of 47 (33/47). The findings indicate that the rate of labor induction was significantly higher in the observation group than in the control group following administration of the combined medication (*P* < 0.05), implying that this result improves the success rate of labor induction, as illustrated in Figure 2.

### 3.8. Comparison of the Incidence of Complications between the Two Groups of Puerperae

The number of parturients who suffered from cervical laceration, postpartum hemorrhage, and cervical edema in the observation group was 2, 1, and 0, respectively, with a complication rate of 5.66%, which was drastically less than that in the control group with corresponding indexes of 5, 5, and 3 and a complication rate of 27.66% (*P* < 0.05), as demonstrated in Table 6.

## 4. Discussion

Clinically, PROM in the third trimester has greater negative effects on both the mother and the infant than in normal pregnancy [17]. Following membrane rupture, pathogenic bacteria in the vagina are susceptible to ascending infection, and the severity of infection is determined by the timing of membrane rupture [18]. Under normal conditions, if the membrane rupture is not treated appropriately and promptly, it is highly likely to induce fetal distress due to oligohydramnios, placental abruption, and umbilical cord prolapse and subsequently lead to neonatal aspiration pneumonia, which poses a serious threat to the fetus's life [19]. Consequently, in clinical practice, if there are no symptoms of labor or the cervix is not developed enough, appropriate therapies could be given to women with PROM at a term greater than 37 weeks to assist them in initiating labor [20].

Prostaglandin preparations and balloon dilation are forbidden when promoting cervical ripening and inducing labor in such women, and only low-dose oxytocin may be used to promote cervical ripening [21]. Oxytocin is a regularly used labor-inducing medication in clinical practice. It works by binding to the oxytocin receptor. While receiving an intravenous infusion of oxytocin to induce labor, the puerpera may suffer irregular uterine contractions, resulting in cervical edema and impeding cervical dilation [22]. Numerous studies have also indicated that oxytocin alone is ineffective as a treatment since it takes a long time to induce labor. Furthermore, many women are unable to bear extended painful uterine contractions, lengthy labor, cervical edema, or cervical damage and thus abandon vaginal trial labor, increasing the rate of cesarean section [23]. As a result, to further test the effect of oxytocin and to find a more appropriate labor induction strategy, we examined the effects of oxytocin alone and the effects of oxytocin and phloroglucinol in combination in women with PROM to discover which was more effective. The Bishop score is a scoring standard for determining cervical ripeness, which can predict whether or not a woman is ready to give birth and the anticipated timing of vaginal delivery [24]. We first evaluated the Bishop score and therapeutic efficacy of two groups, finding that the two indexes of the observation group were significantly higher after drug administration than those of the control group, indicating that the combined treatment may enhance cervical ripening in the first place. Then, we compared the labor process and the success rate of labor induction between the two groups, which revealed that the overall labor stages of the observation group were shorter compared to the control group, with the first stage of labor being the most evident and showing the most significant differences between the two groups. Furthermore, the success rate of labor induction was significantly higher in this group. Our findings suggested that the combination of medications used in our study could effectively relieve cervical spasm, minimize cervical edema, enhance cervical dilatation, shorten the labor phase, and increase the success rate of labor induction. The rationale for this is that phloroglucinol can effectively relieve irregular uterine contractions generated by intravenous oxytocin during labor induction, prevent cervical spasm and damage, and decrease maternal cervical edema [25]. Thus, it was concluded that phloroglucinol in combination with oxytocin could effectively promote regular uterine contractions and cervical canal flattening, stimulate cervix dilation, promote cervical dilation, accelerate cervical ripening, shorten labor, and improve the success rate of labor induction.

Following that, our findings on delivery methods revealed that the vaginal delivery rate of women in the observation group was significantly higher than that of women in the control group, indicating that a combination of medications may be beneficial in increasing the vaginal delivery rate of women. The explanation for this is that once phloroglucinol enters the body, it acts directly on the smooth muscle of the genitourinary tract without having an anticholinergic impact. Additionally, when smooth muscle spasms are relieved, anticholinergic adverse effects such as hypotension or an elevated heart rate are avoided. When taken with oxytocin, it has the potential to boost the therapeutic effect, promote quick cervix ripening, and raise the rate of natural childbirth [12]. The final neonatal result and the incidence of complications indicate that the overall incidence of adverse pregnancy outcomes and complications was significantly lower in the observation group than in the control group, indicating that combination treatment was more safe. This is mostly due to the fact that phloroglucinol has no effect on normal uterine smooth muscle contraction and will not result in a prolonging of the second stage of labor, postpartum uterine atony, or postpartum hemorrhage in most cases. The medicine will not produce unfavorable maternal effects such as high blood pressure, rapid heart rate, uterine rupture, or neonatal asphyxia [26]. On the other hand, phloroglucinol can effectively alleviate puerperium pain and lessen the probability of electing for a cesarean section due to fear of pain; additionally, due to the accelerated delivery process, it can help reduce the incidence of fetal distress, neonatal asphyxia, and puerperium infection with increased security [27].

To summarize, the use of phloroglucinol in combination with oxytocin intravenous infusion during the process of promoting cervical ripening and induction of labor in women with PROM at term can assist women in speeding up cervical dilation, improving the cervical Bishop score, shortening the total labor process, and improving vaginal delivery. Its high success rate and safety profile make it an excellent candidate for clinical advancement and application. However, this study has certain shortcomings and limitations. For instance, certain restrictions apply to sample selection. While the screening was conducted following applicable criteria, it remains questionable whether the specimens chosen are reasonable. Additionally, because the number of samples is small and the research period is limited, clinical research can be expanded with additional time, hence increasing the accuracy of the research results.

## Figures and Tables

**Figure 1:** Comparison of the mode of delivery between two groups of women. Note: ^∗^ means *P* < 0.05.

**Figure 2:** Comparison of success rate of labor induction between two groups of parturients. Note: ^∗^ means *P* < 0.05.

**Table 1:** A comparative analysis of general data [*n* (%)].

Factors	Observation group *n* = 53	Control group *n* = 47	t/X^2^	*P*
Age (years old)			0.107	0.744
≥27	31(58.49)	29(61.70)		
<27	22(41.51)	18(38.30)		
BMI(kg/m^2^)	25.98 ± 1.23	25.88 ± 1.24	0.405	0.686
Average Gestational age			0.170	0.680
≥41	26(49.06)	25(53.19)		
<41	27(50.94)	22(46.81)		
Times of pregnancy			0.076	0.783
≥2	20(37.74)	19(40.43)		
<2	33(62.26)	28(59.57)		
Fetal position			0.058	0.810
Normal	43(81.13)	39(82.98)		
Abnormal	10(18.87)	8(17.02)		
Premature rupture of membrane time (*h*)			0.001	0.990
≥12	27(50.94)	24(51.06)		
<12	26(49.06)	23(48.94)		

**Table 2:** Comparison of the Bishop scores between two groups prior to and following the drug administration.

Time	Observation group *n* = 53	Control group *n* = 47	t	*P*
Before administration	3.14 ± 0.34	3.1 ± 0.23	0.498	0.680
After administration	7.82 ± 0.36	6.06 ± 0.28	27.04	<0.001

**Table 3:** Comparison of the therapeutic effects of two groups.

Therapeutic efficacy	Observation group *n* = 53	Control group *n* = 47	*X* ^2^	*P*
Markedly effective	32(60.38)	22(46.81)	—	—
Effective	19(35.85)	12(25.53)	—	—
Ineffective	2(3.77)	13(27.66)	—	—
Effective rate	51(96.23)	34(72.34)	11.15	<0.001

**Table 4:** Comparison of labor process between two groups (min).

Labor duration	Observation group *n* = 53	Control group *n* = 47	*T*	*P*
First stage of labor	420.78 ± 13.99	616.95 ± 12.01	74.75	<0.001
Second stage of labor	103.11 ± 10.8	104.06 ± 8.2	0.490	0.625
The third stage of labor	15.23 ± 1.09	15.47 ± 1.02	1.132	0.260

**Table 5:** Comparison of the incidence of adverse pregnancy outcomes between two groups.

Incidence of adverse pregnancy outcomes	Observation group *n* = 53	Control group *n* = 47	*t*	*P*
Fetal distress	2(3.77)	6(12.77)	—	—
Neonatal asphyxia	3(5.66)	7(14.89)	—	—
The overall incidence of adverse pregnancy outcomes	5(9.43)	13(27.66)	5.606	0.018

**Table 6:** Comparison of the incidence of complications between the two groups of puerperae.

Adverse reactions	Observation group *n* = 53	Control group *n* = 47	*X* ^2^	*P*
Cervical laceration	2 (3.77)	5 (10.64)	—	—
Postpartum hemorrhage	1 (1.89)	5 (10.64)	—	—
Cervical edema	0	3 (6.38)	—	—
Incidence of complications	3 (5.66)	13 (27.66)	8.970	0.003

## Data Availability

The labeled dataset employed for supporting the achievements of this research is accessible from the corresponding author upon request.
